The article "A Survival Status Classification Model for Osteosarcoma Patients Based on E-CNN-SVM and Multisource Data Fusion" was published in 2022. Journal: Comput Intell Neurosci.

# A Survival Status Classification Model for Osteosarcoma Patients Based on E-CNN-SVM and Multisource Data Fusion

**DOI:** 10.1155/2022/9464182

**Published:** 2022-07-09

**Authors:** Qiang Zhang, Peng Peng, Yi Gu

**Affiliations:** School of Artificial Intelligence and Computer Science, Jiangnan University, Wuxi, Jiangsu 214122, China

## Abstract

Traditional algorithms have the following drawbacks: (1) they only focus on a certain aspect of genetic data or local feature data of osteosarcoma patients, and the extracted feature information is not considered as a whole; (2) they do not equalize the sample data between categories; (3) the generalization ability of the model is weak, and it is difficult to perform the task of classifying the survival status of osteosarcoma patients better. In this context, this paper designs a survival status prediction model for osteosarcoma patients based on E-CNN-SVM and multisource data fusion, taking into full consideration the characteristics of the small number of samples, high dimensionality, and interclass imbalance of osteosarcoma patients' genetic data. The model fuses four gene sequencing data highly correlated with bone tumors using the random forest algorithm in a dimensionality reduction and then equalizes the data using a hybrid sampling method combining the SMOTE algorithm and the TomekLink algorithm; secondly, the CNN model with the incentive module is used to further extract features from the data for more accurate extraction of characteristic information; finally, the data are passed to the SVM model to further improve the stability and classification performance of the model. The model has been demonstrated to be more effective in improving the accuracy of the classification of patients with osteosarcoma.

## 1. Introduction

Cancer [1], also known as malignant tumors by the medical profession, is the result of abnormal cell growth. There are more than 100 types of cancer. Although the types and clinical characteristics of these cancers vary, they have the following commonalities: (1) they are detected late, and patients who are in the middle or late stages when diagnosed account for the majority of the overall cancer diagnosis; (2) the current cancer treatment methods include multiple excision of the malignant tumor, radiotherapy, and chemotherapy. This process will bring great pain to the patient. Osteosarcoma [2], as a type of cancer, has a low incidence rate of only 3 per million, or 2 per 1,000 of the total number of all cancers. However, the degree of malignancy is quite high and the patients are mostly children and adolescents [3]. The cell turnover and growth rate of these people are faster than others, so the cancer cells will grow faster too and the possibility of cure is lower. Early symptoms of osteosarcoma are skeletal pain [4] and unexplained fractures, so they are misdiagnosed as growing pains caused by a body that is growing too fast, delaying the best chance of treatment, which in later stages can develop into severe pain and abnormalities in most organs of the body.

With the development of modern biomedicine, a very close link between osteosarcoma and genes has been discovered through a large number of investigations and studies [5], which makes it possible to treat patients with osteosarcoma precisely based on genetic data. Copy number variation [6] data refer to the reordering of the genome from its original base and can occur in small gene fragments ranging from 1 kb to large gene fragments of several MB. Single nucleotide polymorphisms (SNPs), deletions, insertions and duplications of gene fragments, and variation at multiple loci are the reasons why copy number variation occurs. Its mechanism is the mispairing of two highly homologous DNA sequences on the genome during meiosis or mitosis, resulting in the appearance of a sequence deletion or duplication. The article “The impact of copy number variants on clinical staging and drug resistance mechanisms in osteosarcoma multiforme” suggests that copy number variation is one of several genetic abnormalities that manifest in osteosarcoma. DNA methylation [7] refers to the process of making gene expression different from the original result without modifying the original sequence order of the DNA. Under the influence of DNA methyltransferase, the base pair located in the DNA sequence changes the connection mode of S-adenosylmethionine from a double covalent bond to a single methyl group. The article titled “Research Progress on the Relationship between DNA Methylation and Osteosarcoma” shows that the methylation of various genes is closely related to the staging, diagnosis, metastasis, and prognosis of osteosarcoma. Compared to DNA sequencing data, RNA sequencing [8] data are more sensitive and accurate in detecting fusion genes, which are one of the driving genes for osteosarcoma. In summary, copy number variation data, DNA methylation data, RNA expression data, etc., are all very closely related to osteosarcoma. Their combined analysis is of great importance for the early diagnosis of osteosarcoma, the analysis of the severity of the disease, the establishment of prognostic models, and the assistance of doctors in accurate treatment.

With the development of next-generation gene-sequencing technology [9], the accuracy of the sequencing results has been greatly improved and the types of sequenced genes have become more comprehensive. The use of machine learning methods to establish a survival model and a prognosis model for patients with osteosarcoma can be used as a means of adjuvant therapy to help doctors formulate a more effective and targeted diagnosis and treatment plans and ultimately achieve the purpose of precise treatment [10]. However, the development of gene-sequencing technology also brings some problems to model training. The data dimension is much higher than before. However, there are not many genes that are highly related to diseases. This problem can be described as a dimensional disaster. How to select the genetic data highly related to this disease from the high-dimensional genetic data are a challenge in the current biomedical field. Manual operations and processing based on statistical methods will miss some key genes, and the final result will lead to an inaccurate analysis of the survival status of cancer patients.

With the development of artificial intelligence techniques [11] in the past decades, machine learning [12] as a branch of artificial intelligence has been extremely widely used in many fields, such as image processing, natural language processing, assisted medical diagnosis, and web recommendation systems. The use of machine learning techniques to analyze gene expression data has become one of the most important tools to achieve the goal of precision medicine. However, machine learning faces two challenges in processing gene expression data from osteosarcoma patients: (1) the high dimensionality of the data, which reaches over twenty-four thousand dimensions, is much larger than the number of samples. The redundant and unimportant gene features are removed and suppressed to motivate the important features, which are of considerable importance for predicting the survival status of patients. (2) The amount of data is small, with less than eighty samples of data. In this context, if the model is too complex it will produce an overfitting phenomenon, showing a high classification accuracy in the training set but a low accuracy in the test set. (3) The amount of data between samples of different categories is extremely unbalanced [13], which ultimately leads to falsely high accuracy, low recall, and serious errors in identifying categories with a small number of samples.

Data dimensionality reduction [14] means eliminating unimportant features and retaining important features to improve data quality and enhance model classification. It can be divided into two main categories: feature selection and feature extraction. The former is based on prior knowledge, calculation algorithm results and statistical algorithm results, etc., to filter from original features, and select features that have a great impact on the results. For example, IL1B, IL1RN, IL8, IL10, IL17, and other genes have been confirmed to be highly correlated with gastric cancer [15]. When reducing the dimensionality of gastric cancer gene data, these gene features can be directly selected as the features after dimensionality reduction. The latter method of data dimensionality reduction is different from the former method. Feature extraction needs to change the feature space of the original data and combine different features according to the relationship between the features to obtain the features after dimensionality reduction. The main methods are principal component analysis [16] (hereinafter referred to as PCA) and so on. The PCA algorithm is a linear, global, unsupervised dimensionality reduction algorithm that is implemented by projecting the original data into a new coordinate system, followed by a projection into a *k*-dimensional space, with *k* being the number of features that ultimately need to be retained. The variance in the projection direction is used as a criterion, the larger the variance, the higher the dispersion range. Due to the characteristics of its algorithm, the number of features will be strictly smaller than the number of samples after the dimensionality reduction of the samples using the PCA algorithm. The number of samples is too small, which means that the PCA algorithm cannot obtain an effective projection space, which affects the dimensionality reduction effect and finally makes it difficult for the trained model to show strong classification ability. It can be seen that the rare disease data set represented by osteosarcoma is not suitable for dimensionality reduction using the spatial projection algorithm represented by the PCA algorithm. In this paper, the random forest algorithm is used to first reduce the dimensionality of copy number abnormal data, DNA methylation data, RNA gene sequencing data, and RNA homolog sequencing data individually and then fuse the data according to equal weights.

In recent years, with the development of convolutional neural network [17] (referred to as CNN), many problems that cannot be solved by human computing power alone can be solved with the help of CNN. CNN is a network inspired by the structure of the human neural network. Convolutional neural networks have a wide range of applications including but not limited to computer vision, natural language processing, medical diagnosis, and other fields. Compared with the traditional neural network, the difference is that the convolutional neural network has a convolution layer and a downsampling layer, which can automatically perform feature extraction and transfer the feature-extracted data to the corresponding classifier for classification processing. However, CNN has certain limitations. It uses the convolution kernel to perform convolution calculation on the data, which can only obtain the local receptive field and does not consider the relationship between features from a global perspective. Inspired by SENet [18], the algorithm used in this paper adds an excitation module to the convolutional neural network. Recalculating the weights of different channel features, suppresses the influence of unimportant features and enhances the role of important features. By fully comparing the characteristics of different algorithms and the characteristics of the osteosarcoma gene dataset, this paper will use E-CNN to further extract the features after dimension reduction.

As a kind of machine learning, a support vector machine [19] (SVM for short) has better performance in small sample binary classification and stronger generalization ability compared with other machine learning algorithms. Different from the working principle of the CNN algorithm, SVM is aimed to find an optimal hyperplane between different categories through geometric calculation and uses the hyperplane as the boundary between the categories to complete the classification work. In addition, SVM can also map the data to a higher-dimensional space through kernel functions such as radial basis functions (RBF) and then solve the classification problem of linear inseparable data. As a classifier, SVM has a strong ability to perform binary classification of datasets with small data volumes and low dimensionality. The osteosarcoma gene sequencing data has a small amount of data, but its dimensionality is relatively high. The output data after initial feature selection by random forest [20], followed by deeper feature extraction using a pretrained E-CNN model, satisfies the characteristics of small data volume and low dimensionality described in the previous section. Therefore, this paper uses SVM to replace the Sigmoid activation function of the convolutional neural network as the final classifier, which can further improve the generalization ability and stability of the model.

Ho et al. proposed a model combining principal component analysis (PCA) and convolutional neural network (CNN) to predict the survival status of patients with gastric cancer by analyzing their RNA-seq data [21]; Liu et al. used a combination of a stacked autoencoder and a convolutional neural network model to expand the data using a stacked autoencoder, followed by the analysis of the patient's RNA-seq data using a CNN to classify the type of cancer [22]; Rukhsar et al. [23] used to convert the one-dimensional RNA-seq data into two-dimensional image data, perform zero-completion operations on the edge data and then expand the data using flip, rotate, etc. Then, commonly used networks for processing images, such as ResNet, were used to process the converted image data and thus achieve the function of classifying the survival status of cancer patients.

Copy number variation, DNA methylation data, RNA gene sequencing data, and RNA homologue sequencing data all have varying degrees of impact on the prognosis of cancer patients, but the algorithms described previously only use RNA-seq data for classification studies and do not combine these data for analysis; secondly, these algorithms only use CNN or ResNet, which can only obtain local receptive field and do not consider the relationship between different channels and are prone to overfitting; then secondly, due to the computing mechanism of the PCA algorithm they use, the dimensionality of the data after dimensionality reduction is required to be strictly smaller than that of the sample data, which will inevitably lead to some key genetic data being eliminated. In addition to this, there is an imbalance of data between the different categories of the medical genetic dataset, and these algorithms do not equalize the dataset, which can lead to inflated and unreliable final results.

In this context, this paper proposes a survival status classification model for osteosarcoma patients based on E-CNN-SVM and multisource data fusion. In this paper, an extensive literature review was conducted to fully investigate the impact of copy number variation data, DNA methylation data, RNA gene sequencing data, and RNA homologue sequencing data on osteosarcoma patients, and the four types of data were each reduced in dimension using a feature selection algorithm called a random forest, and then the data were fused with equal weights in the form of data concatenation. Embedding an excitation module in the CNN model to calculate weights based on the importance of features before they are passed to the fully connected layer, to enhance the role of important and weaken the role of unimportant features. In terms of binary classification, SVM shows extremely strong classification performance for samples with a small sample size and low dimensionality. In this paper, we combine both E-CNN and SVM. SVM is trained with data after E-CNN feature extraction to further improve the classification ability and generalization ability of the model.

## 2. Data Acquisition

In this article, 65 patients with osteosarcoma were downloaded from the TargetOS database, a globally recognized and authoritative cancer database. These 65 cases include (1) clinical data on osteosarcoma patients over 3 years, whether the patient died, whether the disease recurred, and whether the cancer cells metastasized. (2) Copy number variation data for osteosarcoma patients, the number of its dimensions per patient is 60,447. (3) DNA methylation data for osteosarcoma patients. The number of its dimensions per patient is 385,292. (4) RNA gene sequencing data for osteosarcoma patients, the number of its dimensions per patient is 59,956. (5) RNA homozygous sequencing data for osteosarcoma patients, the number of its dimensions per patient is 201759. The clinical characteristics of the 65 patients are shown in Table 1.

## 3. Related Work

The algorithmic model devised in this paper fully considers the characteristics of the high-dimensional, unbalanced and small number of gene sequence data sets of osteosarcoma patients, and fully investigates copy number variation (CNV for short), DNA methylation, RNA gene sequence (RNA- Seq-Gene for short), RNA isoform sequence (RNA-Seq-Ios for short) data characteristics, and their respective impact on the survival status of patients with osteosarcoma.

The flowchart of the algorithm is shown in Figure 1 and Table 2. Firstly, the random forest algorithm was used to reduce the dimensionality of the four different aspects of the gene sequencing dataset described in the previous section, followed by fusion of the data with equal weights and then normalization. In addition, the data are balanced by the combination of SMOTE algorithm and the TomekLink algorithm. The SMOTE algorithm uses the upsampling method to expand the samples of the category with a smaller number of samples so that the number of samples of the two categories is consistent; secondly, the TomekLink algorithm is used to clean overlapping samples and edge samples between classes to prevent overfitting during model training. The preprocessed data were divided into a training set and a test set in the ratio of 8 : 2. Due to the small amount of data, the validation set is not divided separately. The five-fold cross-validation method is used to divide the training data into five equal parts, and one of the data is used as the validation set in turn, and the remaining 4 data are used as the training set.

After initial dimensionality reduction, normalization, and partitioning of the data into test and validation sets, the data are secondly subjected to further feature extraction using a convolutional neural network incorporating an excitation module to further improve the quality of the data. Inspired by the SENet neural network, weights are calculated for each feature using the excitation module before the data are fed into the fully connected layer, multiplying the weights with the features and secondly adding them to the unweighted features. Feature weighting fusion through the stimulus module suppresses the effect of unimportant features and enhances the effect of important features. In this paper, we first use the processed data to train the E-CNN model for multiple rounds to optimize the model parameters and save the E-CNN model with the best classification results. When training the E-CNN model, the model is prone to overfitting due to the small number of osteosarcoma samples. In this paper, the early stop algorithm is used to avoid this problem during training, and the model parameters with the smallest rounds of the validation set error function value are saved as the final model parameters when parameter iterations are performed. After the E-CNN model is trained, deeper feature extraction is performed on the data using its input layer to the fully connected layer. The data that has been feature extracted by the E-CNN model is passed into the SVM to train the SVM model, followed by classification using the trained SVM model.

### 3.1. Random Forest

Random Forest is one of many high-performance machine learning algorithms. Because of its high classification accuracy, not easy to overfit, strong antinoise ability, fast training speed, and high tolerance to outliers in data sequences, it has a wide range of applications in economics, geography, and medicine. The Random Forest algorithm is an integrated learning algorithm consisting of several decision trees, based on the Bootstrap sampling method, which selects *M* batches of data from unprocessed source data multiple times, randomly and with putbacks, and uses these *M* batches to build *M* decision trees. A single decision tree is built as an embodiment of the greedy algorithm. First, the impurity of each feature is calculated using the Gini coefficient (as shown in (1)) or the information entropy (as shown in (2)) as an evaluation metric, the lower the impurity, the more suitable the feature is as a branch node in the decision tree. Each time, the node with the lowest impurity is selected from the unselected features, and the above-given operation is repeated several times in the remaining nodes until the Gini coefficient is less than a threshold or there are no features to continue building the decision tree.

(1) $$\begin{array}{c} \text{Gini}=1-\sum_{k=1}^{N}P_{k}^{2}\sqrt{b^{2}-4ac}. \end{array}$$

Here, *P*_*k*_ is the proportion of the *k*-th category of samples to the total number of samples *N*.

(2) $$\begin{array}{c} H\left(D\right)=-\sum_{k=1}^{c}p_{k}{\text{log}}_{2}{}^{p_{k}}. \end{array}$$

Here, *D* is the data set, *c* is the total number of categories, *p*_*k*_ is the number of samples in a category, and *k* is a proportion of the total number of samples.

For classification, the random forest uses each batch of data to train a classification decision tree and takes the output of the *M* classification trees with the largest weight as the classification result of the random forest. For the regression task, the random forest uses each batch of data to train a regression tree, and the output of these *M* regression trees is summed and divided by *M* as the final output of the entire random forest. Compared with a single model or one of the parametric models, the classification and prediction capabilities of the random forest are significantly improved, overcoming the problems of overfitting and low accuracy of a single decision tree, as shown in Figure 2.

Currently, the most widely used algorithm for dimensionality reduction is the PCA algorithm, but due to the limitations of the algorithm, the number of features retained after dimensionality reduction must be strictly smaller than the number of samples. Therefore, when the PCA algorithm reduces the dimensionality of the data with a small number of samples, although some noises are removed, some important features are also removed at the same time. It can be seen that the small sample data set represented by osteosarcoma is not suitable for using this algorithm as a dimensionality reduction algorithm. When performing classification and regression tasks, the random forest will determine the importance of each feature based on its contribution to the building of these decision trees. The features with the highest contribution are selected and retained after feature extraction. Because of the properties, it exhibits in dimensionality reduction, the random forest algorithm is used as the dimensionality reduction algorithm in this paper.

### 3.2. SMOTE+ TomekLink

Machine learning is a data-based discipline. When performing classification tasks, where the amount of sample data varies significantly between categories, the classification performance of the trained model can be severely affected, resulting in its false accuracy and low recall. There are two methods for resolving data imbalance: oversampling and undersampling, with the SMOTE algorithm [24] belonging to the former and the TomekLink [25] algorithm to the latter. The algorithm flow of the SMOTE algorithm is shown in Figure 3. The SMOTE algorithm is used to generate new samples for classes with relatively small sample sizes and put them back into the dataset. In this way, the classes with smaller sample sizes are expanded, and thus the data is balanced between the samples of different classes. The algorithmic process is as follows:

(1) Using the Euclidean distance as a criterion, draw m samples from a relatively small number of categories, and denote these m samples as {*X*_1_, *X*_2_, *X*_3_, *X*_4_, *X*_5_,……*X*_*m*−1_, *X*_*m*_}
(2) Based on the idea of the nearest neighbor node algorithm, for each node *X*_*i*_∈, {*X*_1_, *X*_2_, *X*_3_, *X*_4_, *X*_5_,……*X*_*m*−1_, *X*_*m*_}, compute the k nearest neighbor nodes of each sample *X*_*i*_, denoted as *X*_*i*(*pg*)_
(3) Select several samples from *X*_*ik*_, denote them as *X*_*i*(*pg*)_ and generate a random number *c*, where *c* > 0 and *c* < 1, to synthesize a new sample according to the following equation:
  (3) $$\begin{array}{c} X_{\text{new}}=X_{i}+r\text{and}\left(0,1\right)*\left(X_{i\left(pg\right)}-X_{i}\right). \end{array}$$
(4) Place the newly synthesized new sample *X*_new_ into the original dataset

However, using SMOTE as an oversampling technique to equalize the data can lead to the following problems: (1) SMOTE only focuses on the category with a small number of samples but does not take into account the relationship between the two categories, which can lead to the new composite samples crossing the category boundaries. (2) The new samples are generated by merging the samples at the original category boundary as the center, which will blur the category boundary and reduce the quality of the data and eventually lead to the classification model not being able to calculate an appropriate hyperplane. In this paper, we use TomekLinks, an undersampling method, to solve these problems caused by the use of a single SMOTE. The idea of the TomekLink algorithm is as follows: select some sample pairs (*X*_*i*_, *X*_*j*_), where *X*_i_ is the category with a larger number of samples and *X*_*j*_ is the category with a smaller number of samples, and note that, the distance between the two samples is *d*(*X*_*i*_, *X*_*j*_), if there is no *X*_*k*_, satisfying *d*(*X*_*i*_, *X*_*k*_) < *d*(*X*_*i*_, *X*_*j*_), then (*X*_*i*_, *X*_*j*_) is a pair of TomekLinks pair. When performing data cleaning, both pairs are removed from the sample data.

### 3.3. E-CNN

#### 3.3.1. Introduction to CNN

A convolutional neural network (CNN) is a feed-forward neural network that simulates the way human nerves work and was designed by HUB et al. CNN evolved from multilayer perceptrons (MLP for short). Compared with MLPs, CNNs have features such as weight sharing and local sampling. In recent years, CNN has been used extensively in the fields of image, sound, and medicine. The core parts of the CNN network involved in this article are described as follows:

1. *Convolutional Layer*. The convolution layer, the most important part of the entire CNN, uses convolutional kernels (also known as filters) to perform convolutional calculations on the data, a process that involves the extraction of features from the input data. The weights of each kernel do not change during the convolutional computation, which is the weight-sharing property of CNN. The result of the convolutional computation is then output to the next layer through a nonlinear activation function. In this paper, the ReLu activation function is used.
2. *Dropout Layer*. During the training of a neural network, overfitting can occur due to the depth of the network or the small amount of data. The result is locally optimal, but not for the whole. The result is that the model has poor classification performance and does not perform well in the classification task. The Dropout layer randomly discards some weights in each training batch according to preset parameters, which can effectively avoid overfitting and improve the robustness of the model.
3. *Fully C onnected Layer*. Each nerve in the fully connected layer is connected to a neuron in the previous layer, and in this way, the features output from the previous layer are aggregated.

In this paper, a shallow convolutional neural network was designed, which mainly consisted of an input layer, two convolutional layers, two Dropout layers, and two fully connected layers, taking into full consideration the characteristics of the small number and high dimensionality of the osteosarcoma gene data after equal weight fusion. The CNN model designed in this paper is shown in Figure 4(a).

#### 3.3.2. Introduction to Squeeze-and-Excitation Network

The CNN algorithm has the advantages of weight sharing and automatic feature extraction, but it uses convolutional kernels to obtain only local perceptual fields and does not take into account the correlation between the overall features. The core module of SENet is the Squeeze-and-Excitation (SE) module, which uses the degree of influence of a feature on the result as a criterion to recalculate the weights of different channel features to strengthen the effect of features with high influence and weaken the effect of features with low influence. This module is not a complete network structure, but a module for processing data that can be embedded in other network structures. The SE module algorithm flow is as follows:

(1) *Squeeze (Sequence)*: aggregates data within the same channel to form a multidimensional statistic containing only interchannel correlations. This is achieved by global average pooling (GAP). For example, the original data *U* has dimension *H* × *W* and is compressed along its spatial dimension to give the statistic *Z* ∈ *R*^*c*^, by which the *i*-th element of the compressed *Z*_*i*_ can be obtained.
  (4) $$\begin{array}{c} Z_{i}=F_{sq}\left(u_{i}\right)=\frac{1}{H\times W}\sum_{p=1}^{H}\sum_{q=1}^{W}u_{i}\left(p,q\right), \end{array}$$
where *u*_*i*_(*p*, *q*) are the *p* row and *q* column elements passed into the SE module.
(2) *Excitation*: the excitation process is achieved through two fully connected layers. The role of the first fully connected layer is to compress the vector from *X* dimensional to *X*/*C* dimensional, followed by a call to the ReLu activation function; the role of the second fully connected layer is to restore the vector to *X* dimensions, followed by a call to the Sigmoid activation function, whose calculation process is shown in the following equation:
  (5) $$\begin{array}{c} s=F_{ex}\left(z,W\right)=\partial \left(g\left(z,W\right)\right)=\partial \left(W_{2}\delta \left(W_{1}z\right)\right). \end{array}$$
The sigmoid activation function is denoted as *∂*(·), the ReLu activation function expression is denoted as *δ*(·), the parameters of the two fully connected layers are denoted as *W*_1_ ∈ *R*^(*C*/*r*)×*C*^ and *W*_2_ ∈ *R*^*C*×(*C*/*r*)^, the value of *r* is determined by the model performance requirements and the computational complexity, and the generated *s* are the weights of the channels.
(3) *Scale*: the weights *S* represent the importance of each feature through the excitation process. The final output *X*_new_ is obtained by multiplying the weights *S* and the unweighted data *U* after convolution, as shown in equations (6) and (7).
  (6) $$\begin{array}{c} X_{c}=F_{\text{scale}}\left(u_{c},s_{c}\right)=s_{c}u_{c}, \end{array}$$
  (7) $$\begin{array}{c} X_{\text{new}}=\left[X_{1\text{new}},X_{2\text{new}},\ldots ,X_{\text{inew}},\ldots ,X_{\text{cnew}}\right]. \end{array}$$

After the SE module calculation, the weight relationship between the channels after the CNN convolution calculation can be obtained. By multiplying the unweighted data with the weights, the performance of the features with high importance is amplified and the performance of the unimportant features is suppressed. The result is a model that can be effectively enhanced without adding much computing power.

#### 3.3.3. Introduction to the E-CNN Model

The main application of SENet is in the field of image classification, where the image data needs to be flattened before recalculating the individual feature weights, for example by compressing the original spatial dimension of *H* × *W* to 1 × 1 × *C*. The sequencing data of the osteosarcoma gene after equal-weight fusion is itself flattened data, so there is no need to compress the original data before performing the stimulation operation. Inspired by the SE module, an E-CNN neural network model was designed to further improve the classification performance of the model by considering the relationship between each gene feature as a whole and efficiently extracting features from the sequencing data. The E-CNN neural network and CNN neural network are shown in Figure 4.

### 3.4. SVM

Support Vector Machine (SVM) is a high-performance supervised machine learning algorithm with stable classification performance, high interpretability, and generalization ability. The SVM works as follows: let the data set be *T*, the hyperplane be *M*, and the minimum geometric distance between *T* and *M* be *r*. When the value *r* is maximum, then this hyperplane is the optimal hyperplane, and the optimal hyperplane is used as the criterion for classification.

Because of its good results in small sample binary classification, the RBF kernel-based SVM is used as a classifier in this paper. The parameter setting of the SVM affects the heaviest classification performance, and the penalty factor *C* directly affects the choice of the classification boundary. The RBF kernel function is shown in the following equation:

(8) $$\begin{array}{c} K\left(x,x_{i}\right)=e^{\left(-{\left\|x-x_{i}\right\|}^{2}/2\delta \right)}. \end{array}$$

In equation (8), *δ* is the width of the RBF; ‖*x* − *x*_*i*_‖ is the distance between the selected point and the centroid.

## 4. Analysis of Experimental Results

### 4.1. Experimental Environment

All experiments in this article are run on a computer with Intel Xeon(R) CPU E5-2640 v4@2.40 GHz*∗*40 and 64-bit Linux operating system. The compilation software was PyCharm (PyCharm Community Edition 2020.2.2 x64).

### 4.2. Model Parameter Settings

The parameters of the E-CNN-SVM model proposed in this paper are shown in Table 3.

### 4.3. Evaluation Indicators

In the binary classification problem, as shown in Table 4, if the original category of data is death, the number of data correctly predicted to be in the category of death is labeled TP and the number of data incorrectly predicted to be in the category of survival is denoted FN; if the original category of data is survival, the number of data correctly predicted to be in the category of survival is denoted TN and the number of data incorrectly predicted to be in the category of death is denoted FP. To show the advantages of the algorithm in this paper, it will be compared with other algorithms in terms of accuracy (ACC), recall (Recall), *F*1 score(*F*1), and variance (variance).

Accuracy is a measure of the classifier's classification performance; the higher the accuracy, the better the classification performance of the classifier, and is calculated as shown in the following equation:

(9) $$\begin{array}{c} \text{ACC}=\frac{\text{TP}+\text{TN}}{\text{FP}+\text{FN}+\text{FP}+\text{FN}}. \end{array}$$

The recall is how many positive samples are correctly identified and shows the find-all rate of the classifier. The higher the recall, the more accurately the classifier identifies positive example samples, calculated as shown in the following equation:

(10) $$\begin{array}{c} \text{Recall}=\frac{\text{TP}}{\text{TP}+\text{FN}}. \end{array}$$

The precision rate is the number of samples correctly detected as dead as a proportion of all samples predicted as dead by the model. The *F*1 score takes into account both the precision and recall of the classifier, with the precision rate calculated as shown in equation (11) and the *F*1 score calculated as shown in equation (12).

(11) $$\begin{array}{c} \text{Precision}=\frac{\text{TP}}{\text{TP}+\text{FP}}, \end{array}$$

(12) $$\begin{array}{c} F1=2\times \frac{\text{Precision}\times \text{Recall}}{\text{Precision}+\text{Recall}}. \end{array}$$

The variance represents the stability of the model; a smaller value of variance means a more stable model; conversely, a less stable model. The variance calculation formula is shown in the following equation:

(13) $$\begin{array}{c} \text{Variance}=\frac{1}{n}\sum_{i=1}^{n}{\left(x-x_{i}\right)}^{2}. \end{array}$$

In equation (13), *n* is the number of experiments, *x* is the average of the accuracy of the *n* rounds of experiments, and *x*_*i*_ is the accuracy of the *i*-th round of experiments.

### 4.4. Comparison of Evaluation Results

All experiments performed in this paper used a subset of the same osteosarcoma gene sequencing dataset, and the data were processed consistently. Firstly, the random forest algorithm is used for feature selection to reduce the dimensionality of the data, and secondly, the SMOTE algorithm is combined with the TomekLink algorithm to equalize the amount of data between the different categories and to clean the edge data. A random selection of 20% of the data was used as the test set, followed by a five-fold cross-validation approach using the remaining data, with four of the data rotated as the training set and one as the validation set, to avoid overfitting during the training process.

To validate the performance of the proposed E-CNN-SVM multisource data fusion-based survival status classification model for osteosarcoma patients in this paper, the experiments are designed from the following two perspectives as well as comparative experiments: (1) under the same algorithm, the classification results of the model trained with single-source data are compared with those of the model trained with multisource fused data. (2) The algorithm adopted in this paper is compared with the rest of the algorithms under the condition that the models are all trained using multisource fused data.

#### 4.4.1. Data Source Comparison Experiments

E-CNN-SVM, E-CNN, and CNN were used as the experimental models for this subsection. First, the models were trained and tested using four single sources of data: copy number variation data, DNA methylation data, RNA gene sequencing data, and RNA homologous isoform sequencing data, respectively. Secondly, the data fused with equal weights from these 4 data were used for training and testing. The test results of the same model trained with different source data were compared. The experimental results of the E-CNN-SVM model are shown in Table 5, the experimental results of the E-CNN model are shown in Table 6, and the experimental results of the CNN model are shown in Table 7.

From the experimental results in Tables 5–7, it can be seen that the multi-source fusion data integrated copy number variation data, DNA methylation data, and RNA gene sequencing data related to osteosarcoma, resulting in an improvement of the individual models in all directions. The accuracy, recall, *F*1 score, and variance of the same model after training with multiple sources of data were all better than those after training with single-source data.

#### 4.4.2. Model Comparison Experiments

The results of the data source comparison experiments in the previous section have shown that the ability of the models trained using multiple sources of fused data is better than that of the models trained using single-source data. Therefore, in the model comparison experiments, the models were trained using multisource fused data. To illustrate the effectiveness and feasibility of the E-CNN-SVM model used in this paper, it was chosen to be compared with the existing paper models E-CNN model, CNN model, SVM model, XGBoost model, and CNN-LSTM model. The experimental results are shown in Table 8.

From the experimental data in Table 8, we can learn that the E-CNN-SVM model proposed in this paper obtains a better result in terms of accuracy, recall, *F*1 score, and variance. Its performance is much higher than the comparison model in this paper, showing the high performance, robustness, and stability of the E-CNN-SVM model rejected in this paper.

## 5. Conclusion

1. An E-CNN-SVM classification algorithm based on multisource feature homofusion is proposed. The copy number abnormal data, DNA methylation data, RNA gene sequencing data, and RNA homologue sequencing data of osteosarcoma patients were weighted and fused to predict the survival status of patients for classification. The accuracy, recall, and *F*1 score of the predictive classification reached 100%, which is significantly more accurate than other methods for predicting the survival status of osteosarcoma patients and is extremely important for achieving precise treatment of osteosarcoma patients.
2. The features of each channel are weighted by the calculation of the stimulus module before being fed into the fully connected layer of the CNN model, which can significantly improve the feature extraction capability of the CNN model.
3. The equal-weight fused data is again subjected to deeper feature extraction with the parameter-optimized E-CNN model and then fed into SVM for classification, which has higher accuracy than simply using E-CNN and SVM.
4. Although the algorithm in this paper exhibits strong properties, its generalization capability cannot be validated due to the relatively small dataset, which is a pain point in the whole field of medical analysis. The dataset will certainly be expanded from different aspects in the future to enhance the generalization ability of the model.

## Figures and Tables

**Figure 1:** The flow chart of the E-CNN-SVM and multisource algorithm.

**Figure 2:** The random forest construction process.

**Figure 3:** Schematic diagram of the SMOTE algorithm for constructing new nodes.

**Figure 4:** The schematic diagram of CNN & E-CNN. (a) The schematic diagram of the CNN model. (b) The schematic diagram of the E-CNN model.

**Table 1:** Clinical characteristics of these patients.

Clinical features	
Number of cases	65

Age at illness (years)	15.09 ± 4.89

Gender	
Male	36
Women	29

Race	
White people	39
Black people	10
Asian	7
Unknown	9

Primary site	
Lower limbs	59
Pelvis	2
Upper limb	4

Survival time (days)	1339.31 ± 982.08

**Table 2:** The steps of the E-CNN-SVM and multisource algorithm.

Step 1	The copy number variation data, DNA methylation data, RNA gene sequencing data, and RNA homologue sequencing data are each reduced in dimension using the random forest algorithm
Step 2	Equal weighted fusion of these four types of data
Step 3	Combine the SMOTE algorithm with the TomekLink algorithm to clean and equalize the data
Step 4	Pretrain the E-CNN model and save the optimal model
Step 5	Feature extraction of data using the input layer to the fully connected layer of the E-CNN model
Step 6	Use the processed data to train the SVM model and use the trained model for classification

**Table 3:** The E-CNN-SVM model parameters.

CNN		
First convolutional layer	Filters: 128	kernel_size: 1
First dropout layer	Rate: 0.3	
Second convolutional layer	Filters: 64	kernel_size: 1
Second dropout layer	Rate: 0.3	
Motivation module	Compression ratio: 4	
Fully connected layer	Units: 2	

SVM		
Penalty factor	0.9	
Cache_size	3000	
Kernel	rbf	

**Table 4:** Confusion matrix.

Patient survival status	Classificationpredicted as death	Category predictionfor survival
Death	TP	FN
Survival	FP	TN

**Table 5:** E-CNN-SVM experimental data.

Number	Model	Data type	Accuracy (%)	Recall (%)	*F*1 score (%)	Variance
1	E-CNN-SVM	Multisource	100	100	100	0
2	E-CNN-SVM	Copy number variation	100	100	100	0
3	E-CNN-SVM	DNA methylation	100	100	100	0
4	E-CNN-SVM	RNA-seq-gene	100	100	100	0
5	E-CNN-SVM	RNA-seq-Ios	92	75	86	0

**Table 6:** E-CNN experimental data.

Number	Model	Data type	Accuracy (%)	Recall rate (%)	*F*1 score (%)	Variance
1	E-CNN	Multisource	97	97	96	0.0015
2	E-CNN	Copy number variation	79	69	69	0.0036
3	E-CNN	DNA methylation	86	76	77	0.0031
4	E-CNN	RNA-seq-gene	82	71	78	0.0105
5	E-CNN	RNA-seq-Ios	88	88	84	0.0012

**Table 7:** CNN experimental data.

Number	Model	Data type	Accuracy (%)	Recall rate (%)	*F*1 score (%)	Variance
1	CNN	Multisource	86	97	81	0.0031
2	CNN	Copy number variation	75	69	66	0.0036
3	CNN	DNA methylation	80	74	74	0.0041
4	CNN	RNA-seq-gene	79	71	73	0.0036
5	CNN	RNA-seq-Ios	83	75	80	0.0054

**Table 8:** Model comparison experimental data.

Number	Model	Data type	Accuracy (%)	Recall rate (%)	*F*1 score (%)	Variance
1	E-CNN-SVM	Multisource	100	100	100	0.0000
2	E-CNN	Multisource	97	97	96	0.0015
3	CNN	Multisource	86	97	81	0.0031
4	SVM	Multisource	76	35	51	0.0081
5	XGBoost	Multisource	76	66	64	0.0065
6	CNN-LSTM	Multisource	59	0	0	0.0000

## Data Availability

The dataset used to support the findings of this study are available from the corresponding author upon request.
